# An ROI Extraction Method of Finger Vein Images Based on Large Receptive Field Gradient Operator for Accurate Localization of Joint Cavity

**DOI:** 10.1155/2022/9231637

**Published:** 2022-05-30

**Authors:** Huimin Lu, Yifan Wang, Weiye Liu, Yupeng Li, Jingfeng Ning

**Affiliations:** School of Computer Science and Engineering, Changchun University of Technology, Changchun 130102, China

## Abstract

Region of interest (ROI) extraction is a key step in finger vein recognition preprocessing. The current method takes the finger region in the vein image as the ROI, but this method cannot obtain better recognition accuracy because it only removes the background noise of the image and ignores factors such as the position and shape of the finger. To solve this problem, we limited the ROI to a fixed region between two finger joint cavities, proposed a new large receptive field gradient operator, and designed and implemented a new method for ROI extraction. It uses a large receptive field to search the target, which is similar to human vision, thus solving the problem of difficult ROI localization for images with large gradient areas. Moreover, for external factors such as noise and uneven illumination in the vein image, the interference factors can be eliminated by averaging them to a larger range with a larger size operator to improve the accuracy of the subsequent matching recognition. To verify the effectiveness of the proposed method, we conducted sufficient matching experiments on three public finger vein datasets. On various datasets, our method significantly reduced the identified EER value, with the lowest EER value reaching 0.96%. The experimental results show that the proposed ROI extraction method can effectively eliminate the influence of finger position, finger shape, and other factors on the subsequent recognition performance, accurately locate the finger joint cavity, and effectively improve the recognition performance.

## 1. Introduction

Finger vein recognition is a biometric recognition technology that uses near-infrared light to collect finger vein images and identify them according to the extracted finger vein features [1]. Compared with common biometric features such as face [2] and fingerprint [3], the biggest advantage of finger vein feature is that it is located inside the human body. Moreover, due to the convenience of collection and quick identification of digital vein information, the identification can only be done in vivo, and it has a high level of safety [4]. After years of development, finger vein recognition has been widely used in smart homes, intelligent transportation, education examinations, intelligent security, and other fields. In recent years, with the global COVID-19 pandemic, serious international health security issues have emerged, and there is an urgent need for a convenient and secure identification method. As a second-generation biometric technology, finger vein recognition has gained wide attention due to its high level of convenience and security [5]. It is noteworthy that noncontact and unconstrained finger vein recognition technology can achieve high recognition accuracy. Therefore, it can realize identification while providing safety guarantees for public health. However, noncontact and unconstrained digital vein image acquisition will inevitably introduce various factors that affect recognition performance to a greater extent, such as uneven light, finger deformation, and displacement. If we use the finger region as the ROI and only remove the noise in the image background, we cannot solve the influence of finger deformation, displacement, and other factors on recognition performance. Therefore, it is necessary to design and develop a more robust and effective ROI extraction method for finger vein images to minimize the impact of these factors on recognition performance. In the study of existing joint cavity localization methods, we found that it is unreasonable to only search the joint cavity locally. The greyscale variation in the joint cavity is a large gradient, and its region usually occupies a large part of the finger region. For human vision, it is impossible to find the joint cavity if it is only observed in a small field of view. For computers, similar to human vision, the vertical orientation of the ROI is often inaccurate if only a local region is searched. The existing methods are usually pixel counting for the local area or localization based on the unstable features of the joint cavity region. In this way, the shape and position of the finger, as well as the noise generated by the device, strongly affect the positioning of the joint cavity, resulting in incorrect or unstable position information. We propose a large receptive field gradient operator, which can accurately locate the joint cavity, further segment the finger region, limit the area between the two joint cavities of the finger, and eliminate the influence of finger displacement and deformation. Each search covers approximately 20% of the finger region, and the noise in the image is greatly reduced due to the use of a large field operator. In addition, we study the size of the gradient operator of a large receptive field in detail to find the optimal size. The main contributions of this paper are as follows:

1. A novel gradient operator called the large receptive field gradient operator is proposed, which can solve the problem of joint cavity localization caused by a large gradient in the process of finger joint cavity imaging.
2. According to the change in finger joint cavity width, we designed the most suitable range of receptive fields for the localization search of finger joint cavities in finger vein images so that the size of the large receptive field gradient operator is most suitable for the localization of finger joint cavities.
3. A new ROI extraction method for finger vein images is proposed. It consists of three steps: first, the finger region is extracted by the Kirsch operator and dynamic threshold based on the 3*σ* criterion; second, the proposed large receptive field gradient operator is used to locate the joint cavity position as a vertical reference line, and then the finger region is further segmented; third, the ROI of the finger vein image is obtained through vertical lines and some soft finger features.

The organizational structure of this paper is as follows: Section 2 reviews the representative research results of ROI extraction in recent years; Section 3 introduces the ROI extraction method combining the Kirsch operator with the dynamic threshold strategy of 3*σ* criterion; Section 4 elaborates on the proposed joint cavity localization method, that is, the large receptive field gradient operator; Section 5 describes a large number of experiments designed and carried out based on three different public finger vein datasets to test and verify the recognition performance of the proposed method; and Section 6 clarifies the research conclusions of this paper and prospects the future research direction of ROI extraction filed.

## 2. Related Work

ROI extraction is a part of image preprocessing and an important part of finger vein recognition. The quality of ROI extraction directly affects the effect of image enhancement and normalization. Generally, the steps of ROI extraction include horizontal reference line localization, image correction, and vertical reference line localization. According to different localization methods, ROI extraction is divided into threshold-based methods and mask-based methods.

The threshold-based method is a kind of method widely used in the early research of finger vein recognition. Such methods usually use a fixed threshold or OTSU threshold. After obtaining the binary finger image, we use it as a mask to remove the background image. Kumar and Zhou [4] obtained a binary image using a fixed threshold of 230, subtracted it from the binary image using a horizontal Sobel operator, and finally obtained the mask through connected domain analysis. P. Gupta and P. Gupta [6] binarized the image using the global threshold, obtained the finger region through morphological operation, and used it as a mask. Threshold-based methods have rarely been used in recent research. Ideally, the pixel values in the finger region are higher or lower than those in the background region. However, in practical applications, due to the different lighting conditions of different acquisition devices, it is difficult to avoid the pixel value distribution in the finger region being similar to that in the background region.

Masked-based methods are the most widely used. Generally, this type of method uses the horizontal edge extraction operator to extract finger edges and remove the complex background in the image. Lee et al. [7] divided the image into upper and lower parts and used the horizontal edge detection operator to extract finger edges. Wang and Tang [8] combined the horizontal operator in [7] with the horizontal Sobel operator to detect finger edges and remove line segments whose length is less than the threshold. Finally, only the edges of the finger are retained in the binarized image. Inspired by [7], Lu et al. [9] extended the horizontal Prewitt operator to extract finger edges and corrected the wrong edges using finger orientation angles. Song et al. [10] used the Laplace operator to extract finger edges and used average curvature to complete finger edges. In the process of detecting finger edges with a horizontal edge extraction operator, the maximum response value is usually used as the finger edge. Most operators are sensitive to noise data. As the background difference of vein images acquired by different devices is relatively large, it is easy for operators to take background noise as the maximum response, resulting in the detection of incorrect edges. Therefore, this type of method usually requires more postprocessing operations [11]. Yao et al. [12] first introduced the Kirsch operator to the edge extraction of finger vein images and extracted edges using two horizontal Kirsch operator templates. They also set three dynamic thresholds, combined with the 3*σ* principle, for further processing finger edges. Tao et al. [13] used the Mask RCNN method to predict the ROI mask. Wang et al. [14] used the active contour model (ACM) to obtain the finger vein ROI mask. Gao et al. [15] proposed simplified statistical region merging (SSRM) to obtain finger regions, and a new directed link clustering method (DLCM) and parameter selection (PS) were introduced to ensure edge qualification and further correct the tilt angle. This method is very effective for finger edge detection, which can extract weak finger edges and filter out background noise to a large extent.

The purpose of ROI extraction of finger vein images is to quickly extract the same region from the same finger vein image collected under different conditions. After obtaining the horizontal segmentation reference line for the ROI from the inner tangent of the finger edge, the problem focuses on how to find the appropriate segmentation reference line in the vertical direction to limit the ROI to a fixed region of the finger. Initially, most researchers chose to use a fixed-size window for vertical reference line segmentation. For example, literature [8, 10] used fixed-size rectangular boxes to delineate fingers. After finding the centroid of the binary image, Rosdi et al. [16] used the centroid as the centre of the rectangular box to delineate the finger. Recent studies have paid more attention to the structural characteristics of fingers because the gap between finger cartilage can transmit more near-infrared light, so it appears as two brighter regions at the joint cavities of the collected finger vein images (displayed as higher pixel values on the digital image, as shown in Figure 1). Researchers usually choose the finger joint cavity as the reference line for vertical segmentation and propose some joint cavity search algorithms. The initial algorithm was based on the cumulative value of regional pixels. Literature [17] proposed calculating the cumulative value of pixels per column and then selecting the maximum cumulative value to locate the joint cavity. In the follow-up study, it was found that the uneven illumination of the finger vein capture device affected the search effect of the joint cavity. Therefore, to improve the joint cavity localization method based on the cumulative value of a single column of pixels, the researchers proposed a calculation method of the multicolumn pixel cumulative value based on a sliding window and used the maximum value to locate the finger joint cavity [18]. Qiu et al. proposed a joint cavity search algorithm based on double sliding windows, which uses two windows for difference to eliminate the problem of affecting recognition [19] in the imaging process. Zeng et al. [20] proposed that sliding method summation was employed to reduce missing pixels from finger ROIs. Yang et al. [21] proposed a method in which the finger region was obtained using a fixed window and image standard deviation. Then, the finger region was enhanced using a Gaussian-based anisotropic ordinal filter (GAOF). Finally, the maximum cumulative value in the calculated row was the distal venous joint. After positioning the finger joint cavity, the segmentation reference line in the vertical direction was obtained, and the ROI was extracted from the corrected finger vein image using the obtained horizontal and vertical segmentation reference lines. At this point, the difference in finger vein features between different individuals is relatively the largest, and the difference in finger veins collected by the same individual under different conditions is relatively the smallest, which lays a foundation for the next step of vein image enhancement and improving the final matching and recognition performance. However, the existing articular cavity localization methods mentioned above cannot solve the problem of a large range of grey gradients generated by the joint cavity of the finger vein during imaging. Methods based on pixel accumulation can mostly find the brightest local region, but due to the influence of illumination, the brightest region is usually not the whole joint cavity region. The key to locating the joint cavity is to calculate the gradient in the image. Therefore, we propose a large receptive field gradient operator and a new joint cavity localization method. Using the operator we proposed, a wide range of gradients in the vertical direction of the finger region and more accurate joint cavity localization can be achieved.

## 3. ROI Extraction Combining the Kirsch Operator and the 3*σ* Criterion Dynamic Threshold Strategy

### 3.1. Kirsch Edge Detection

Edge extraction operators have been widely used in ROI extraction [22]. However, there are a series of individuals, environments, devices, and other factors in the acquisition process, resulting in a large number of low-quality finger vein images, especially the disappearance of finger edges or the generation of weak edges, which have a great impact on the extraction of finger edges. When there are a large number of weak edges in an image, the usual edge detectors cannot obtain the complete edge or introduce a large number of false edges. The Kirsch edge operator achieves excellent performance in identifying weak edges and false edges [12]. It uses eight templates (as shown in Figure 2) to convolve the image. Usually, only two templates (M1; M2) in the horizontal direction are used to extract finger edges, and the gradient with the largest directional response is selected as the edge.

### 3.2. Dynamic Thresholding Based on 3*σ* Criterion

The labelling strategy for the longest connected component in a binary image is a good way to filter finger edges. Using connected components to filter edges is in line with practical application scenarios, and it provides higher real-time performance and robustness. For the Kirsch edge detector, setting different thresholds produces different edge images. High thresholds are used to detect clearly defined edges, and correspondingly, low thresholds provide more complete weak edges. Additionally, different regions of the same vein image have different qualities; thus, different thresholds are needed. Yao found that, under ideal conditions, when performing edge detection [12], there are only finger edges in the binary image. Considering this, the greyscale distribution in Kirsch gradient images can be regarded as a Gaussian distribution. In a Gaussian distribution, the mean *μ* determines the location of the overall distribution. A variable that is closer to the mean is considered to have a higher probability of occurrence. The variance in the variable *σ* determines the amplitude of the distribution. The smaller the variance is, the more concentrated it is, and vice versa. The 3*σ* criterion in the Gaussian distribution can process samples with near-Gaussian distributions. For the 3*σ* criterion, different interval values are distributed with different probabilities, which are (*μ* − *σ, μ* + *σ*): 0.6827, (*μ* − 2*σ, μ* + 2*σ*): 0.9544, and (*μ* − 3*σ, μ* + 3*σ*): 0.9974 (as shown in Figure 3).

In [9], the image processing method based on Gaussian bilateral filtering was first used, which divided the image into four parts: upper left corner, lower left corner, upper right corner, and lower right corner. Dynamic thresholds are set according to the 3*σ* criterion. The initial threshold is set to *µ* + 2*σ,* and only 2.28% of the points are reserved as edges. In this case, distinct strong edges are preserved for high-quality images. For weak edges that are not detected, the threshold can be released to *µ* + *σ*, extending the candidate edges to 15.87%. Finally, those edges that still do not satisfy the requirements should be filtered out using *μ* + 0.5*σ*. During the detection process, the length of the connected components is used to automatically determine whether further processing is needed. An edge larger than the threshold *L* (generally 1/2 of the width of the detection area) is considered to be a relatively complete edge. If the connected component is less than *L*, the threshold needs to be released for further processing. Finally, the four subgraphs are integrated, the complete edge line is completed by interpolation, and the complex background noise is removed by the edge line.

Usually, this type of method removes the complex background noise, but the finger position and shape information remain in the ROI. However, in the subsequent vein pattern matching, the position and shape of the fingers do not determine the features. These features largely cause the classifier to make incorrect judgements. In response to this problem, we further divide the finger region by limiting the ROI between the two joint cavities to remove the position and shape information of the finger in the ROI. Moreover, we propose a new large receptive field gradient operator to accurately locate the joint cavity.

## 4. Large Receptive Field Gradient Operator

In some datasets, there is little difference between image samples of the same finger; that is, there is little variation in the sample data within the class. The methods in [12] can achieve high recognition accuracy for the extraction of the ROI of such datasets, but we found that this type of method only uses the finger region to extract the ROI, which often requires a stable and unchanged finger position and finger shape. Once the position and shape of the finger change greatly, the performance of the system identified by the ROI obtained by these methods will decline sharply. Therefore, the large receptive field gradient operator we proposed is necessary. After obtaining the coordinates of the finger, the image is corrected, the finger region is further segmented by the proposed method, and the ROI region between the proximal and distal joint cavities is limited, which can eliminate the influence of the changes in the position and shape of the finger on the recognition system performance.

In the study of the existing joint cavity localization methods, we found that only positioning the joint cavity is often inaccurate. Similar to human vision, the greyscale change in the joint cavity is a larger gradient, and its area usually occupies a large portion of the finger area. If only observed in a small range, it is impossible to determine whether this joint cavity is located. Similarly, for computers, the vertical orientation of the ROI is often inaccurate if only local areas are searched. Thus, this paper proposes a method for searching the joint cavity based on a large receptive field, with each search covering approximately 20% of the finger region:

1. Reduce the finger area to a quarter of the original image using “double triple” interpolation to obtain *g*′(*x*, *y*) of size (*m*′ × *n*′).
2. Use our proposed new large receptive field (6 × 7) gradient operator (Figure 4) to extract the vertical gradients from finger vein images.
3. Select the location of the distal joint cavity and use *j*_*r*_, *j*_*l*_  to indicate the position of the distal and proximal joint cavities, respectively, then calculate the cumulative value of pixels in each of the three columns in gradient plot *g*′ and denote them as *S*_*c*_, and then use formula (1) to obtain the coordinates of their minimum value; after reduction, this is the position of the distal joint cavity, which is multiplied by 3 and 4 to determine the reduction gradient of the pixel value statistics and the position change generated when the image size is reduced. In addition, the position of the proximal joint cavity is obtained using the width *w* of the finger at the distal joint, where 1.25 refers to the ratio of the length of the interarticular cavity to the width of the distal finger joint cavity obtained in statistics [23]:

(1) $$\begin{array}{c} \;\left\{\begin{array}{c} S=\sum_{i}^{m^{\prime }}g^{\prime }\left(i,c:c+3\right),\;c=1,4,7,\ldots ,n^{\prime }-3\\ j_{r}=\arg\min\left(S\right)*3*4\\ j_{l}=j_{r}-1.25*w \end{array}\right). \end{array}$$

The complete process of ROI extraction is described as follows: first, the finger edge is obtained by using the finger region extraction method in reference [12] (as shown in Figure 5(a)), and the minimum inner tangent of the finger is used as the segmentation reference line in the horizontal direction (as shown in Figure 5(b)); second, the finger edge midline is fitted, the angle between the finger and the horizontal direction is obtained as the correction angle, and the image is corrected by affine transformation; third, the finger region of the corrected image is segmented by the horizontal segmentation line; then, the large receptive field gradient operator proposed in this paper is used to locate the joint cavity, and the segmentation reference line in the vertical direction can be obtained. To ensure minimal loss of feature information in the ROI, we update the horizontal segmentation line twice. In the first case, the coordinates of the corrected finger edge change, so the horizontal reference lines also change accordingly. We choose to use formula (2) to update the coordinates of the reference line. In the second case, we limit the selection of horizontal reference lines to two joint cavities. Similarly, we use formula (2) to update the horizontal reference line (the final reference segmentation line is shown in Figure 5(c)). Finally, we use horizontal and vertical reference lines to delineate the ROI on the corrected image (as shown in Figure 5(d)).

(2) $$\begin{array}{c} \left\{\begin{array}{c} \text{u}p^{\prime }=\text{up}-2*\varphi \\ {\text{lower}}^{\prime }=\text{lower}-2*\varphi \end{array}\right). \end{array}$$

Figure 6 shows the original ROI obtained using our proposed method and the corresponding vein features extracted using the maximum curvature [24] method. By comparing the ROI obtained in literature [12] with the method proposed in this paper, it can be found that the ROI extraction method limited to the area between the two joint cavities of the finger can effectively remove the position and shape information of the finger so that there is almost no difference in the characteristics between the same finger samples. In each ROI, we retain only the unique vein information of each finger, which is the most important and effective vein information of each finger. Then, after size normalization and feature extraction, there is only the vein pattern of the finger in the ROI image, which can maximize the performance of the recognition system.

## 5. Experimental Results

### 5.1. Datasets

In some published finger vein datasets, there are few interclass changes in the vein data samples representing the same finger. Therefore, the robustness of some ROI extraction and recognition methods has not been verified in practice, and accurate matching and recognition cannot be realized in practical applications. For the experiments in this paper, we selected three publicly available finger vein datasets: UTFVP [25], published by the University of Twente in the Netherlands, MMCBNU_6000 [26], published by Korea Joensuu University, and FV-USM [27], published by University Technology Malaysia. Among them, the UTFVP dataset is characterized by smaller interclass differences and less background noise for clear finger vein images, while the MMCBNU_6000 dataset and FV-USM dataset are characterized by larger sample sizes and sufficient interclass differences for the same finger vein data. In particular, in the FV-USM dataset, each finger was captured 6 times in one acquisition, and each finger participated in two acquisitions over a period of two weeks to generate more practical data samples. The details of these three datasets are shown in Table 1.

### 5.2. Dimension of Gradient Operator with a Large Field of View

#### 5.2.1. Required Height and Width

The gradient operator in a large field of view solves the grey change in the gradient type by calculating the grey area of the image, which takes more calculation time. We solve this problem by reducing the size of the image, but we still need to obtain the best efficiency while ensuring accuracy when we locate the ROI. Therefore, by changing the size of the gradient operator in the large field of view and comparing them, we obtain different equal error rates (EERs) on the FV-USM dataset (as shown in Table 2). It should be noted that when the width of the operator is 3, each row is calculated using [1, 0, −1]. When the width of the operator is greater than 3, we fix the scanning area of the finger joint cavity to a width of 3 pixels, such as [1,…, 1, 0, 0, 0, −1,…, −1], and then the subsequent increase in width only needs to add 1 and −1 at both ends of the operator. The template matching method for obtaining EER is described in detail in Section 5.3. When using the conventional gradient scale (3 × 3) operator, a larger EER value (3.048) was obtained, and within a certain range, the EER value obtained from the matching experiments gradually decreased with increasing operator length and width. Through the experiment, we concluded that when the size of the operator is 6 × 7, the lowest EER value of 2.811 was obtained.

Figure 7 shows a heatmap of the EER values calculated by operators of different sizes. It can be clearly observed that when the width of the operator increases gradually, EER values show a significant downward trend. In addition, for operators with smaller widths, the EER values obtained are more stable when the width increases. This is because the robustness of the gradient operator with a small range to noise is relatively poor, while the risk of noise influence is relatively small when the gradient operator is in the large field of view. For the FV-USM dataset, we obtained a more stable EER value at a width of 7 and a minimum EER value (2.811) at a height of 6. This is because the size of the finger joint cavity is limited, and oversizing will cover the finger area at both ends of the joint cavity, resulting in an incorrect gradient calculation.

#### 5.2.2. Appropriate Joint Cavity Width

In finger vein imaging, the joint cavity region presents a gradual greyscale, but there is a more obvious grey mutation at the end of the joint cavity close to other structures in the finger. We can find the most appropriate width value of the finger joint cavity by constantly changing the size of the region in the gradient operator when scanning the joint cavity.  Table 3 shows the different EERs obtained under different joint cavity detection widths, where 1, 3, 5, and so on represent the number of zeros in each row of the operator.  Table 3 shows that, for the joint cavity regions in the gradient operator that are not involved in the gradient calculation, a width that is too small will lead to a gradient calculation error, while a width that is too large will waste calculation resources and affect performance. When the width is large enough, nonjoint cavity regions affecting the localization accuracy will be covered. Therefore, when using a smaller joint cavity detection area, a larger EER (3.082) is obtained. When the joint cavity detection area is maintained at 5–11 pixels, the EER is stable at 2.913, and with the continuous increase in width, the calculation efficiency gradually decreases, and the error further increases. The minimum EER (2.811) value is obtained when the size of the operator is 6 × 7 and the joint cavity detection area is 3.

### 5.3. Matching

#### 5.3.1. Comparison of Different ROI Methods

To more intuitively verify the effectiveness of our proposed method, we used the maximum curvature [24] method and repeated line tracking [28] method to extract features and carry out template matching [29] experiments. For the similarity measurement in template matching, we chose to use the correlation coefficient method. We first used Yao's method and our proposed method to obtain the ROI, followed by feature extraction and then comparative experiments, and used the false acceptance rate (FAR) and false rejection rate (FRR) to evaluate the matching performance. Due to different thresholds, different FARs and FRRs are obtained. When FAR and FRR are equal, the value is equal to the error rate (EER).  Figure 8 shows the ROC curves obtained from the matching experiments, and Table 2 demonstrates the EERs for all experiments.

According to Figure 8 and Table 4, the effectiveness of our method can be further verified by analysing the experimental results. When collecting finger vein information, the finger position information and shape information are not the key features required for subsequent matching and recognition but interfere with the performance of matching and recognition. Because our ROI extraction method effectively removes interference information such as finger position and shape, the EERs of our method are the lowest. It can be seen that the ROI obtained by further processing the finger region can have better robustness. Specifically, on the FV-USM dataset, our method shows more obvious advantages. Moreover, when we further process the finger region, the EERs of the matching experiment decrease significantly, which is more consistent with the practical application. It should be noted that we propose an ROI extraction method without in-depth study of other factors affecting the matching performance in the subsequent feature extraction process. It is believed that we can obtain more ideal matching accuracy by carefully adjusting the parameters of the feature extraction algorithm.

#### 5.3.2. Comparison of Different Localization Methods of Joint Cavity

In the previous section, we verified the necessity of further finger segmentation, but if the joint cavity localization is not accurate, it may lead to worse results. Therefore, in this experiment, some representative localization methods of the joint cavity of the finger vein image are compared with the localization method of the large receptive field gradient operator we proposed, including (1) the single sliding window method [18], (2) the fixed-window method [8], (3) the double sliding window method [19], and (4) the single-line cumulative value method [17]. Similarly, we use the method in literature [12] to segment the finger region and obtain a horizontal reference line. Then, the horizontal reference line is used to segment the finger vein image. Finally, different joint cavity localization methods are used to obtain different ROIs. The maximum curvature method [24] and repeated line tracking method [28] are still used to extract pattern features.

The experimental results presented in Figure 8 and Table 4 show that our method achieved excellent EER on each dataset. After analysing the experimental results of different methods, we found that the fixed-window method always achieved good EERs on different datasets. Therefore, we used our independently developed finger vein collection device to test the fixed-window method. It was found that this method only performs well on open datasets with little image variation. When we collect with our device, if we add some changes in the direction, position, and other factors of the finger, the EER value of this method increases dramatically. The single-slide window method and the single-row pixel accumulation method (both calculate pixel values in local columns) tend to look for the “brightest” region in the vein image. However, in practical applications, due to the influence of various external factors, the joint cavity region is not always the brightest region, which will lead to incorrect localization. The double sliding window locates the joint cavity by subtracting the pixels in both windows, which effectively removes noise from the image by the subtraction operation, but it is still essentially a pixel-based operation that does not accurately localize the joint cavity. By observing the ROIs obtained, we found that, due to the inhomogeneity of optical noise and background noise, some low-quality images have obvious joint cavity effects of accurate localization. One of the more important factors is that the joint cavity can produce a large-area grey gradient during the imaging process, and the existing methods cannot solve this problem well. In fact, this is because the existing methods are only statistical pixel gradient methods, which only simply process column pixel values. For this problem, our method can effectively solve it by extracting the gradient of the image in the vertical direction and can obtain a lower EER.

To compare the effects of various methods more intuitively, we conducted visual experimental verification of the localization effects of different joint cavity localization methods on different datasets. Two samples from each dataset were filtered out, and the four different methods were marked with four different colours (cyan: single sliding windows; fuchsia: dual-sliding windows; blue: single line; red: proposed method in this paper).  Figure 9 shows the visualization of different localization methods on different datasets. In Figure 9(a), the three methods for comparison are very sensitive to the change in finger illumination and are mostly located in the brightest area of the finger. However, due to the influence of illumination, the joint cavity is not always the brightest area during imaging, while the method proposed in this paper is always located in the position where the gradient changes the most, that is, the left side of the joint cavity, proving that our method has strong robustness and stability. In Figure 9(b), we observe that, in the finger vein images of this condition, there is a large brighter area in or near the joint cavity, which easily leads to incorrect positioning for the existing localization methods. The reason is that these methods use a smaller search area, which often leads to being limited to this area (the brightest but unstable), whereas the method of this paper has a broader field of vision, can search over a much larger area, and consistently can locate the finger joint cavity on the leftmost side of the joint cavity, which is very stable.  Figure 9(c) shows that there are many complex background noises in the finger vein images, which for unstable upper and lower finger edge detection methods often provide an incorrect search area for joint cavity localization. The single-line and dual-sliding window methods are very susceptible to such problems. However, the experimental results show that the method proposed in this paper is still steadily located on the rightmost side of the joint cavity, which shows that our method is very stable and robust.

## 6. Conclusions

The current representative ROI extraction methods only remove the background noise of the image and only use the finger region to obtain the ROI. However, in ROI extraction, factors such as the movement position and shape of the finger can adversely affect subsequent recognition performance. Therefore, we propose a large receptive field gradient operator. On the one hand, by using this operator, we can effectively solve the problem of a large-scale grey gradient in the imaging process of the joint cavity to realize the accurate localization of the joint cavity. On the other hand, the finger region is further segmented by the obtained vertical reference line, and the ROI is limited between the two finger joint cavities, which effectively eliminates the influence of factors such as finger position and shape on the recognition performance. The experiments on three publicly available datasets show that the ROI obtained by our proposed method has better matching performance. It is more robust and more consistent with practical applications. Currently, the global epidemic has raised the issue of public health security to an unprecedented height, and finger vein recognition will evolve towards contactless and unconstrained acquisition. Additionally, the shape of the joint cavity extraction operator will be further investigated, and with the development of deep learning, it will be a good solution for finger vein ROI localization. In the future, this more robust and efficient ROI extraction method will be very meaningful and valuable for adapting to more complex application scenarios.

## Figures and Tables

**Figure 1:** Finger region pixel distribution.

**Figure 2:** Kirsch operator.

**Figure 3:** The 3*σ* criterion in the Gaussian distribution.

**Figure 4:** Large receptive field gradient operator.

**Figure 5:** The process of robust ROI extraction method of finger vein image proposed in this paper.

**Figure 6:** The effect of extracting ROI using the proposed method and extracting vein features using the maximum curvature method.

**Figure 7:** Heatmap of EER values calculated by operators of different sizes.

**Figure 8:** Comparison of ROCs obtained by different ROI extraction methods.

**Figure 9:** Comparison of different methods of joint cavity localization. (a) MMCBNU_6000. (b) UTFVP. (c) FV-USM.

**Table 1:** Dataset information for experiments.

Datasets	No. of subjects	No. of images	No. of fingers for each subject	No. of images for each subject	Image size
UTFVP	60	3816	6	4	672 × 380 pxl
MMCBNU_6000	100	1440	6	10	640 × 480 pxl
FV-USM	123	6000	4	6	640 × 480 pxl

**Table 2:** EER values obtained by operators of different sizes.

Height	Width								
	3	5	7	9	11	13	15	17	19
3	3.048	2.981	2.879	3.099	3.015	3.015	2.879	2.879	2.879
4	2.933	2.893	2.870	2.982	3.014	3.014	2.911	2.913	2.879
5	3.013	3.014	2.879	2.981	2.913	2.913	2.913	2.879	2.879
6	3.048	3.048	**2.811**	2.947	3.014	2.913	2.947	2.913	2.913
7	2.981	2.947	2.839	2.981	2.947	2.879	2.879	2.947	2.947
8	2.981	3.082	2.851	2.981	2.947	2.879	2.913	2.913	2.913
9	3.048	2.981	3.014	2.981	2.879	2.828	2.845	2.879	2.913
10	3.048	3.014	2.913	3.014	2.981	2.947	2.913	2.879	2.913
11	2.981	2.964	2.879	3.014	3.014	2.947	2.913	2.913	2.879
12	3.150	3.014	3.014	3.014	2.981	2.947	2.947	2.879	2.913
13	3.014	3.048	2.947	3.082	3.082	2.981	2.981	2.879	2.879
14	2.981	3.048	2.879	2.981	3.014	2.981	2.947	2.913	2.913
15	2.947	3.014	2.913	3.082	3.082	3.014	2.947	2.913	2.879

This is the lowest EER and represents the best matching performance. We have added additional descriptions in the paper.

**Table 3:** EERs obtained by different widths of joint cavity detection region.

Joint cavity width	1	3	5	7	9	11	13	15
EER	3.082	**2.811**	2.913	2.913	2.913	2.913	2.947	2.981

This is the lowest EER and represents the best matching performance. In the paper, we describe it (“The minimum EER (2.811) value is obtained when the size of the operator is 6 × 7 and the joint cavity detection area is 3.”).

**Table 4:** EERs calculated by different ROI extraction methods.

Feature	ROI	MMCBNU_6000 (%)	UTFVP (%)	FV-USM (%)
Maximum curvature	Yao's method	6.33	1.39	8.85
	Single sliding window method	6.76	4.24	5.89
	Fixed window	4.97	3.29	2.47
	Dual-sliding windows	5.77	4.51	6.38
	Single-line accumulation	7.19	3.59	4.50
	Proposed method	4.91	2.77	2.81

Repeated line tracking	Yao's method	4.26	1.74	13.22
	Single sliding window method	3.76	1.35	3.59
	Fixed window	2.38	1.04	1.52
	Dual-sliding windows	3.22	1.53	4.84
	Single-line accumulation	3.95	1.12	3.34
	Proposed method	3.73	0.97	1.69

## Data Availability

Previously reported data (UTFVP, MMCBNU_6000, and FV-USM) were used to support this study and are available at (DOI:10.1109/ICB.2013.6612966; DOI: 10.1109/CISP.2013.6744030; DOI:10.1016/j.eswa.2013.11.033). Prior studies (and datasets) are cited at relevant places within the text as references [25–27].
